# Denoising Diffusion MRI via Graph Total Variance in Spatioangular Domain

**DOI:** 10.1155/2021/4645544

**Published:** 2021-12-07

**Authors:** Haiyong Wu, Senlin Yan

**Affiliations:** School of Electrical Engineering, Nanjing Xiaozhuang University, Nanjing 211171, China

## Abstract

Diffusion MRI (DMRI) plays an essential role in diagnosing brain disorders related to white matter abnormalities. However, it suffers from heavy noise, which restricts its quantitative analysis. The total variance (TV) regularization is an effective noise reduction technique that penalizes noise-induced variances. However, existing TV-based denoising methods only focus on the spatial domain, overlooking that DMRI data lives in a combined spatioangular domain. It eventually results in an unsatisfactory noise reduction effect. To resolve this issue, we propose to remove the noise in DMRI using graph total variance (GTV) in the spatioangular domain. Expressly, we first represent the DMRI data using a graph, which encodes the geometric information of sampling points in the spatioangular domain. We then perform effective noise reduction using the powerful GTV regularization, which penalizes the noise-induced variances on the graph. GTV effectively resolves the limitation in existing methods, which only rely on spatial information for removing the noise. Extensive experiments on synthetic and real DMRI data demonstrate that GTV can remove the noise effectively and outperforms state-of-the-art methods.

## 1. Introduction

DMRI is a unique way in the *in vivo* characterization of anatomical connectivity in the human brain [1]. However, it is frequently impeded by pronounced thermal noise due to its echo-planar acquisition strategies and low signal-to-noise ratio (SNR) [2]. One practical way to reduce the noise variance of DMRI data is averaging several acquisitions [3]. Therefore, it requires an extended period that is not suitable for clinical settings. On the other hand, many postprocessing algorithms have been applied in DMRI denoising to improve the data quality. Most of them can be roughly grouped into transform-based and spatial approaches.

Transform-based denoising methods are frequently used in signal processing because it is generally believed that noise and signal are more easily distinguished in the transform domain. Nowak [4] proposed the wavelet domain filter for reducing Rician noise in MRI. This method filters the squared magnitude of MRI in that distribution changes from Rician to noncentral Chi (nc-*χ*). Wood and Johnson [5] proposed an MRI denoised strategy based on the wavelet packet. This method exceptionally performs well on removing Rician noise with low SNR since wavelet packet provides a more compact signal representation than single wavelet decomposition. Other transform-based approaches, including curvelet transform [6] and block-matching and 3D (BM3D) [7] denoising schemes, have been proven to tackle Rician noise in MRI data efficiently.

Spatial denoising methods utilize the neighbor information around the pixel to reduce the variance caused by noise. Henkelman [8] presented the pioneering study on estimating Gaussian noise in MR images and smoothened them by convolution filtering, but this method blurs sharp edges that provide crucial clinical information. Gerig et al. [9] applied nonlinear anisotropic diffusion (AD) filters to 2D and 3D MRI denoising. AD filters can remarkably leverage the MRIs' quality in terms of persevering boundaries. However, AD methods assume that the processed MRI are piecewise constant and the noise is Gaussian distributed with zero means. Both of those mentioned above are not applicable for MRI. Tong et al. [10] proposed an improved AD algorithm that used an adaptive scheme to select parameters to reduce Rician noise in MRI. To avoid tuning numbers of parameters carefully, Awate and Whitaker [11] proposed a nonparametric neighborhood statistics technique for MRI denoising. They inferred the prior from the degraded MRI and the knowledge of the Rician noise model. The uncorrupted MRI statistics are modeled in a nonparametric Markov Random Field (MRF) and estimated by the expectation-maximization algorithm. Experiments show that this method can well preserve important features in brain MRI. Fabio et al. [12] defined a 3D local Gaussian MRF (LGMRF) that allows tuning the filter in an unsupervised way. The LGMRF model can automatically implement the regularization to find the trade-off between noise reduction and detail preservation.

TV-based regularization [13] is one of the most influential denoising algorithms since it can effectively reduce the variance while preserving shape edges. Martin et al. [14] proposed a TV-Rician denoising model for MRI data by solving a semi-implicit numerical scheme. Liu et al. [15] extracted the noise map through a two-step wavelet-domain estimation method, then denoised the MRI data based on a generalized TV model. Later, the authors extended their work by combining none local mean (NLM) filters [16]. The aforementioned methods mainly process the data in the spatial domain (i.e., *x*-space) while ignoring that DMRI data consists of spatial and diffusion wavevector space. These denoising algorithms lead to new smoothing artifacts caused by averaging over differential oriented signals, particularly in the highly curved white matter structures.

Recently, Chen et al. have proposed two novel NLM-based denoise methodologies in joint *x* − *q* space. Before NLM denoising, for each point in *x* − *q* space, they (1) defined a spherical patch from which they extracted the rotation-invariant features patch matching [17] and (2) performed graph framelet transforms to extract robust rotation-invariant features after encoding the *q*-space sampling domain using a graph [18]. Graphs have the ability to well modeling the data with irregular and complex structures [19]. In this paper, we represent the joint *x* − *q* space DMRI data with a graph and associate signal coefficients with graph nodes. Then, we consider the denoising DMRI data on the graph as an optimization problem, which seeks to minimize a TV function based on graph edge signals. The main contribution of our GTV denoising framework includes threefold: (i) the proposed method avoids computing rotation-invariant features; (ii) the minimizing variation procedure harnesses not only over spatial space but also angular space, allowing information to be shared across DW images for effective denoising; (iii) the information in angular space represents structures oriented in different directions, so our method is expected to be more effective for denoising without introducing new artifacts.

The remainder of this paper is organized as follows. We describe the detail of the proposed method in Section 2 and evaluate the effectiveness on synthetic data and public real data in Section 3.  Section 4 shows our further discussion of this work. Finally, we conclude this work in Section 5.

## 2. Method

### 2.1. Graph Representation

Given a graph *G* = (*𝒱*, *w*), where *𝒱* = {*v*_*n*_}_*n*=1_^*N*^ represents the set of *N* nodes and *w* ∈ *ℂ*^*N*×*N*^ is an affinity matrix, which characterizes the relationships between every pair of nodes on graph. The graph signal is a mapping function *𝒱*⟶*ℂ* that associates signal coefficients *S*_*n*_ ∈ *ℂ* to each node *v*_*n*_ ∈ *𝒱* of the graph.

We show how to represent DMRI data using a graph. Specifically, given a sampling point (*i*, *j*) in spatioangular domain, which is determined by a spatial location **x**_*i*_ ∈ ℝ^3^ and a gradient direction **q**_*j*_ ∈ ℝ^3^ and diffusion weighting *b*_*j*_ ∝ ‖**q**_*j*_‖^2^, we consider it as a node of the graph and define the affinity weight with another node (*i*′, *j*′) as [20]

(1) $$\begin{array}{c} w_{i,j;i\prime ,j\prime }≔\exp\left(-\frac{{\left\|x_{i}-x_{i\prime }\right\|}_{2}^{2}}{\sigma_{x}^{2}}\right)\times \exp\left(-\frac{1-{\langle {\overset{\wedge }{q}}_{j},{\overset{\wedge }{q}}_{j\prime }\rangle }^{2}}{\sigma_{q}^{2}}\right)\times \exp\left(-\frac{{\left(\sqrt{b_{j}}-\sqrt{b_{j^{\prime }}}\right)}^{2}}{\sigma_{b}^{2}}\right), \end{array}$$

where *σ*_*x*_, *σ*_*q*_, and *σ*_*b*_ are three parameters controlling the commitments of spatial, angular, and diffusion weight, respectively [21].

### 2.2. GTV of DMRI

We define the GTV of DMRI signal *S* with respect to graph *𝒢* as

(2) $$\begin{array}{c} \underset{\left(i,j\right)}{\sum }{\left\|\nabla_{G}S_{i,j}\right\|}_{1}=\underset{\left(i,j\right)}{\sum }\underset{\left(i^{\prime },j^{\prime }\right)\in N_{i,j}}{\sum }\sqrt{w_{i,j;i\prime ,j\prime }}{\left\|S_{i,j}-S_{i\prime ,j\prime }\right\|}_{1}, \end{array}$$

where *S*_*i*,*j*_ is a diffusion signal associated with spatial location **x**_*i*_, gradient direction **q**_*j*_, and diffusion weighting *b*_*j*_. *𝒩*_*i*,*j*_ is the spatioangular neighborhood of *S*_*i*,*j*_. We set *w*_*i*,*j*;*i*′*j*′_ = 0 where (*i*′, *j*′)∉)*𝒩*_*i*,*j*_; then, (2) becomes the standard *l*_1_-norm ‖∇_*𝒢*_(*S*)‖_1_.

To denoise the DMRI data, we propose

(3) $$\begin{array}{c} \underset{S}{\min}\frac{1}{2}{\left\|S-S^{\prime }\right\|}_{2}^{2}+\lambda {\left\|\nabla_{G}\left(S\right)\right\|}_{1}, \end{array}$$

where the quadratic fidelity term is to force the underlying clean data *S* to stay close to the acquired noisy DMRI data *S*′, and tuning parameter *λ* controls the trade-off between two parts of (3) [22]. Since (1) assumes the nearer nodes have a higher weight, (3) ensures they have lower dissimilarities. It is worth noting that our GTV takes the neighborhood region compared to traditional TV, which only considers the neighbors of a sample along Cartesian axes.

### 2.3. Optimization

Graph gradient ∇*𝒢* is a linear operator (hereafter denoted as *L*) which associates the DMRI signal to the corresponding node, and consequently, (3) is usually referred to the *primal problem* since it can be expressed as the following form:

(4) $$\begin{array}{c} \underset{x}{\min}f\left(x\right)+g\left(Lx\right), \end{array}$$

where *f*(*x*) represents the fidelity term in (3) and it is convex and differential with a *β*-Lipschitz continuous gradient ∇_*f*_(*x*). (4) is related to the following dual problem [23]:

(5) $$\begin{array}{c} \underset{v}{\min}f^{*}\left(-L^{T}v\right)+g^{*}\left(v\right), \end{array}$$

where *f*^∗^ is the conjugate of function *f*. It is worth noting that only a small number of neighbors are taken into account in the proposed graph (i.e., the number of edges is much smaller than that of nodes); therefore, (5) is much easier to solve than (4). The second term *g*(*D*) = *λ*‖*D*‖_1_ where *D* = *L*(*S*) is convex and has proximity operator [24].

(6) $$\begin{array}{c} {\text{prox}}_{\tau ,g}\left(D\right)=\mathrm{sgn}\left(D\right)\circ \max\left(\left|D\right|-\tau \gamma ,0\right). \end{array}$$

Note that *τ* is the step size in the iterative optimization process and is typically set to the inverse of the Lipschitz constant, and ∘ denotes the Hadamard product. With the aid of these tools, we can recover the unique solution of (3) via a forward-backward-based primal-dual algorithm [23, 24].

## 3. Experiments

### 3.1. Datasets

We evaluate the proposed GTV based on a synthetic dataset and a subject from Traveling Human Phantom (THP) that was collected for a multisite neuroimaging reliability study [25]. The research was completed according to the endorsed guidelines.

In order to evaluate the denoising performance of the proposed method for various fiber structures, we use phantom*α*s to produce a synthetic dataset [26]. The fiber geometric configuration is completely identical to that in ISBI 2013 HARDI challenge, and the gradient direction files are consistent with the THP dataset, i.e., using *b* = 1000 s/mm^2^ with a total of 30 noncollinear gradient directions. Image dimensions are 55 × 55 × 55 with 2 × 2 × 2 mm^3^ resolution.

THP data was acquired using the Siemens 3T TrioTim MR scanner with the following imaging protocol: 128 × 128 imaging matrix, 2 × 2 × 2 mm^3^ resolution, TE = 92 ms, and TR = 1,200 ms. *b* values and gradient direction are the same as the synthetic data.

To evaluate the performance of our proposed approach, we add Gaussian distributed noise with zero mean and different deviation of *σ*_*n*_ = 100,200 and 300 to the synthetic data. Some example images are shown in Figure 1.

### 3.2. Parameter Settings

We have implemented Algorithm 1 with the help of open-source Python packages including PyGSP [27] and PyUNLocBox [28], which, respectively, facilitate a number of operations on graph and solvers on nondifferentiable convex optimization problems using proximal splitting methods [29]. The relative tolerance stopping criterion *ε* is set to 10^−3^, and the maximum number of iterations is set to *N* = 200 [24]. Both of them are set automatically by PyUNLocBox. Larger values of tuning parameter *λ* lead to smoother solutions of (3) whereas smaller values emphasize better fitting to the required measurements. Hence, we set *λ* = 0.1.

The proposed approach regards each sampling point in the spatioangular domain as a node. Therefore, DMRI data will lead to a large graph, requiring colossal memory, and GTV is difficult to converge. To overcome this weakness, we construct the graph by dividing the DMRI data into overlapping patches in spatial space, then optimize each patch simultaneously. Although a larger patch can capture more context information, we set the size of the patch to 5 × 5 × 5 and the overlap step to 2 according to our compute unit with 12 GB memory.

As mentioned in (1), construction of the graph involves three parameters: *σ*_*x*_, *σ*_*q*_, and *σ*_*b*_. We normalize each exponent in exponential functions to [0, 1] as it was suggested in [21]. The maximum distance in a 5 × 5 × 5 patch equals to 64, and therefore, we set *σ*_*x*_ = 8. We fix parameters *σ*_*x*_ = 8 and *σ*_*b*_ = 1, then evaluate the influence of parameter *σ*_*q*_ by measures of peak signal-to-noise ratio (PSNR) and structural similarity index (SSIM) [30]. As indicated in Figure 2, the proposed method will achieve the best performance when *σ*_*q*_ = 1.1.

### 3.3. Methods for Comparison

We compared GTV with the following state-of-the-art methods:

1. Adaptive nonlocal means (ANLM): ANLM [31] is an improved version of the NLM algorithm, which is adaptive soft coefficient matching. Based on [31], we set the patch radius to 2
2. Marcenko-Pastur PCA (MP-PCA): MP-PCA [32] classifies the principal components of the observed DMRI signal based on Marcenko-Pastur distribution, then removes them as noise. Both ANLM and MP-PCA are implemented by DIPY [33]
3. XQ nonlocal means (XQ-NLM): XQ-NLM [17] denoises the signal via weighted averaging of self-similar information, which is defined in the spatial-angular domain. The parameters are set to the default values as suggested in [17]

We transform the Rician signal to its Gaussian-distributed counterpart using Özarslan et al.'s method [34]. For a fair comparison, we estimate the nonstationary noise by MP-PCA for ANLM, XQ-NLM, and GTV. Then, we determine the standard deviation of stationary noise via PIESNO [35].

### 3.4. Results

We first quantitatively show the denoise performance through measures including SSIM and PSNR in Figure 3 where the *x*-axial represents the noise level. Although GTV has achieved slightly higher SSIM than MP-PCA and XQ-NLM, all of them are close to 1, meaning that denoised data structures closely resemble the original synthetic data. Regarding PSNR, GTV and XQ-NLM have outperformed MP-PCA and ANLM, which indicates filtering in spatial-angular space can remove more noise.

We randomly select two regions of interest (ROI) marked by red and blue rectangles, respectively. Close-up views of DW images and RMSE maps are presented in Figure 4. The first and third rows of DW images show that MP-PCA, XQ-NLM, and GTV have outperformed ANLM. With the help of RMSE maps in the below rows, we can observe that the reconstruction error of GTV is smaller than MP-PCA and XQ-NLM, which indicates GTV can restore the image more precisely.

One disadvantage of NLM-based methods is that the denoising process may add method noise which usually blurs the outputs. The region marked by the red square in Figure 5 is a part of the boundaries between white matter and the ventricles. Due to the consideration of information in the *q*-space, XQ-NLM and GTV have recovered the edges as MP-PCA does. In contrast, ANLM has removed some noise, but the remaining is far from perfect. The region marked by the blue square in Figure 5 includes a contingent of boundaries, and it shows that GTV reconstructs the internal details while its boundary is the clearest.

Residual maps are used to evaluate whether structural information has been removed after denoising. In Figure 6, residual maps of MP-PCA, XQ-NLM, and GTV have less structure information than that of ANLM. This observation provides evidence that ANLM has lower edge-preserving abilities in Figure 5 from another perspective.

We further evaluated the denoising performances through fiber ODFs. THP [25] is single-shell (with only a single *b* = 0 image) DMRI data. Response functions for single-fiber white matter (WM), as well as gray matter (GM) and cerebrospinal fluid (CSF), were estimated from the denoised data using an unsupervised method [36]. Then, we performed Single-Shell 3-Tissue Constrained Spherical Deconvolution (SS3T-CSD) [37] to obtain WM-like FODs as well as GM-like and CSF-like compartments in all voxels using MRtrix3Tissue, which is a fork of MRtrix3 [38]. The first row in Figure 7 shows a slice of FOD-based directionally encoded color (DEC) maps [39]. The fiber ODFs in the region marked by the red rectangle indicate more coherence after denoising. The region marked by a blue rectangle indicates that the proposed GTV has more effectively reduced spurious fiber peaks that result from noise.

## 4. Discussion

GTV can remove the noise more effectively, which may be attributed to the following aspects:

1. DMRI uses *q*-space information to characterize the direction and scale of the diffusion for water molecules in the tissues. The proposed GTV takes advantage of neighborhood similarity information in the spatioangular domain while constructing a graph
2. Graph representation is a versatile model where nodes are associated with DMRI signal intensity, and edges reflect structural information

Although the proposed algorithm is very effective for denoising, it is not superior to the recent novel DMRI denoising method Patch2Self [40] which denoises DMRI with a self-supervised deep learning strategy. Furthermore, there may be two limitations in this study. First, taking each sample in spatioangular space as an independent node leads to a big graph, which requires a large amount of memory for storing graph properties, including affinity weighted matrix and Fourier basis. It can be relieved by dividing the data into patches [21]. Second, optimization of total variation takes a relatively long time. We speed up the denoising by using the multicore CPUs to optimize each patch simultaneously. Possible solutions include refactoring the software using C++ and combining a two-step optimization approach [16] developed to solve the resulting convex denoising GTV model.

## 5. Conclusion

In this study, we formulated denoising processing as an optimization problem, finding the DMRI data with minimal graph total variation. Both spatioangular information of DMRI data were incorporated to construct the graph, which significantly contributed to this paper. The performances of our proposed method were assessed via experiments on synthetic and real data. Numerical results demonstrate that GTV outperforms various current state-of-the-art approaches in terms of preserving edges and removing noise. Future works may extend GTV to patch GTV that associates values in a patch with a graph node.

## Figures and Tables

**Figure 1:** Some examples of synthetic data degraded by Gaussian noise with different deviations.

**Figure 2:** Selecting of *σ*_*q*_ via indicators including SSIM and PSNR.

**Figure 3:** Quantitative comparison of denoising performance, where *x*-axis represents standard deviation of noise.

**Figure 4:** Regional close-up views of DW images and RMSE maps.

**Figure 5:** Comparison of edge-preserving performances among different denoising algorithms.

**Figure 6:** Residual maps. Representation of whether structural information is removed after denoising.

**Figure 7:** Fiber ODF comparison of various denoising algorithms.

**Algorithm 1:** Forward-backward-based primal-dual for GTV optimization.

## Data Availability

The real data is downloaded from https://openneuro.org/datasets/ds000206/versions/1.0.0/download.

## References

[1] Sporns O., Tononi G., Kötter R. (2005). The human connectome: a structural description of the human brain. *PLoS Computational Biology*.

[2] Kirilina E., Lutti A., Poser B. A., Blankenburg F., Weiskopf N. (2016). The quest for the best: the impact of different EPI sequences on the sensitivity of random effect fMRI group analyses. *NeuroImage*.

[3] Johansen-Berg H., Behrens T. E. J. (2013). *Diffusion MRI: From Quantitative Measurement to In Vivo Neuroanatomy*.

[4] Nowak R. (1999). Wavelet-based Rician noise removal for magnetic resonance imaging. *IEEE Transactions on Image Processing*.

[5] Wood J. C., Johnson K. M. (1999). Wavelet packet denoising of magnetic resonance images: importance of rician noise at low snr. *Magnetic Resonance in Medicine: An Official Journal of the International Society for Magnetic Resonance in Medicine*.

[6] Ma J., Plonka G. (2007). Combined curvelet shrinkage and nonlinear anisotropic diffusion. *IEEE Transactions on Image Processing*.

[7] Dabov K., Foi A., Katkovnik V., Egiazarian K. (2007). Image denoising by sparse 3-d transform-domain collaborative filtering. *IEEE Transactions on Image Processing*.

[8] Mark R., Henkelman (1985). Measurement of signal intensities in the presence of noise in mr images. *Medical Physics*.

[9] Gerig G., Kubler O., Kikinis R., Jolesz F. A. (1992). Nonlinear anisotropic filtering of mri data. *IEEE Transactions on Medical Imaging*.

[10] Tong C., Sun Y., Payet N., Ong S.-H. (2012). A general strategy for anisotropic diffusion in MR image denoising and enhancement. *Magnetic Resonance Imaging*.

[11] Awate S. P., Whitaker R. T. (2007). Feature-preserving mri denoising: a nonparametric empirical Bayes approach. *IEEE Transactions on Medical Imaging*.

[12] Baselice F., Ferraioli G., Pascazio V. (2017). A 3d mri denoising algorithm based on Bayesian theory. *Biomedical Engineering Online*.

[13] Rudin L. I., Osher S., Fatemi E. (1992). Nonlinear total variation based noise removal algorithms. *Physica D: Nonlinear Phenomena*.

[14] Martin A., Garamendi J.-F., Schiavi E. (2013). Mri tv-rician denoising. *International Joint Conference on Biomedical Engineering Systems and Technologies*.

[15] Liu R. W., Shi L., Huang W., Xu J., Yu S. C. H., Wang D. (2014). Generalized total variation-based MRI Rician denoising model with spatially adaptive regularization parameters. *Magnetic Resonance Imaging*.

[16] Liu R. W., Shi L., Yu S. C. H., Wang D. (2015). A two-step optimization approach for nonlocal total variation-based Rician noise reduction in magnetic resonance images. *Medical Physics*.

[17] Chen G., Yafeng W., Shen D., Yap P.-T. (2019). Noise reduction in diffusion MRI using non-local self-similar information in joint x−q space. *Medical Image Analysis*.

[18] Chen G., Dong B., Zhang Y., Lin W., Shen D., Yap P.-T. (2019). Denoising of diffusion MRI data via graph framelet matching in x-q space. *IEEE Transactions on Medical Imaging*.

[19] Ortega A., Frossard P., Kovacevic J., Moura J. M. F., Vandergheynst P. (2018). Graph signal processing: overview, challenges, and applications. *Proceedings of the IEEE*.

[20] Chen G., Yafeng W., Shen D., Yap P.-T. (2016). XQ-NLM: denoising diffusion MRI data via x-q space non-local patch matching. *In Medical Image Computing and Computer-Assisted Intervention (MICCAI)*.

[21] Hong Y., Kim J., Chen G., Lin W., Yap P.-T., Shen D. (2019). Longitudinal prediction of infant diffusion MRI data via graph convolutional adversarial networks. *IEEE Transactions on Medical Imaging*.

[22] Lu W., Duan J., Qiu Z., Pan Z., Liu R. W., Bai L. (2016). Implementation of high-order variational models made easy for image processing. *Mathematical Methods in the Applied Sciences*.

[23] Komodakis N., Pesquet J.-C. (2015). Playing with duality: an overview of recent primal?dual approaches for solving large-scale optimization problems. *IEEE Signal Processing Magazine*.

[24] Mahmood F., Shahid N., Skoglund U., Vandergheynst P. (2018). Adaptive graph-based total variation for tomographic reconstructions. *IEEE Signal Processing Letters*.

[25] Magnotta V. A., Joy T., Matsui D. L. (2018). *DWI Traveling Human Phantom Study*.

[26] Caruyer E., Daducci A., Descoteaux M., Houde J. C., Thiran J. P., Verma R. (2014). *Phantomas: a flexible software library to simulate diffusion MR phantoms*.

[27] Defferrard M., Martin L., Pena R., Perraudin N. (2017). *Pygsp: graph signal processing in python*.

[28] Defferrard M., Pena R., Perraudin N. (2017). *Pyunlocbox: Optimization by Proximal Splitting*.

[29] Combettes P. L., Pesquet J.-C. (2011). Proximal splitting methods in signal processing. *Fixed-Point Algorithms for Inverse Problems in Science and Engineering*.

[30] Wang Z., Bovik A. C., Sheikh H. R., Simoncelli E. P. (2004). Image quality assessment: from error visibility to structural similarity. *IEEE Transactions on Image Processing*.

[31] Coupé P., Manjón J. V., Robles M., Collins D. L. (2012). Adaptive multiresolution non-local means filter for three-dimensional magnetic resonance image denoising. *IET Image Processing*.

[32] Veraart J., Fieremans E., Novikov D. S. (2016). Diffusion MRI noise mapping using random matrix theory. *Magnetic Resonance in Medicine*.

[33] Garyfallidis E., Brett M., Amirbekian B. (2014). Dipy, a library for the analysis of diffusion MRI data. *Frontiers in Neuroinformatics*.

[34] Özarslan E., Koay C. G., Basser P. J. (2009). A signal transformational framework for breaking the noise floor and its applications in MRI. *Journal of Magnetic Resonance*.

[35] Koay C. G., Özarslan E., Pierpaoli C. (2009). Probabilistic Identification and Estimation of Noise (PIESNO): a self- consistent approach and its applications in MRI. *Journal of Magnetic Resonance*.

[36] Dhollander T., Mito R., Raffelt D., Connelly A. (2019). Improved white matter response function estimation for 3-tissue constrained spherical deconvolution. *In ISMRM*.

[37] Dhollander T., Connelly A. (2016). A novel iterative approach to reap the benefits of multi-tissue CSD from just single-shell (+b=0) diffusion MRI data. *In ISMRM*.

[38] Tournier J.-D., Smith R., Raffelt D. (2019). _MRtrix3_ : a fast, flexible and open software framework for medical image processing and visualisation. *NeuroImage*.

[39] Dhollander T., Smith R. E., Tournier J. D., Jeurissen B., Connelly A. (2015). Time to move on: an FOD-based DEC map to replace DTI’s trademark DEC FA. *In ISMRM*.

[40] Fadnavis S., Batson J., Garyfallidis E., Larochelle H., Ranzato M., Hadsell R., Balcan M. F., Lin H. (2020). Patch2self: denoising diffusion MRI with self-supervised learning. *Advances in Neural Information Processing Systems, Volume 33*.

